# Interpretable Machine Learning to Optimize Early In-Hospital Mortality Prediction for Elderly Patients with Sepsis: A Discovery Study

**DOI:** 10.1155/2022/4820464

**Published:** 2022-12-15

**Authors:** Xiaowei Ke, Fangjie Zhang, Guoqing Huang, Aimin Wang

**Affiliations:** ^1^Department of Emergency Medicine, Xiangya Hospital, Central South University, Changsha, 410000 Hunan, China; ^2^National Clinical Research Center for Geriatric Disorders, Xiangya Hospital, Changsha, 410000 Hunan, China

## Abstract

Sepsis-related mortality rates are high among elderly patients, especially those in intensive care units (ICUs). Early prediction of the prognosis of sepsis is critical, as prompt and effective treatment can improve prognosis. Researchers have predicted mortality and the development of sepsis using machine learning algorithms; however, few studies specifically focus on elderly patients with sepsis. This paper proposes a viable model for early prediction of in-hospital mortality among elderly patients diagnosed with sepsis. We extracted patient information from the Medical Information Mart for Intensive Care IV database. We employed several machine learning algorithms to predict the in-hospital mortality of elderly ICU patients with sepsis. The performance of the model was evaluated by using the AUROC and *F*1 score. Furthermore, the SHAP algorithm was used to explain the model, analyze how the individual features affect the model output, and visualize the Shapley value for a single individual. Our study included 18522 elderly patients, with a mortality of 15.4%. After screening, 59 clinical variables were extracted to develop models. Feature importance analysis showed that age, PO2, RDW, SPO2, WBC, and urine output were significantly related to the in-hospital mortality. According to the results of AUROC (0.871 (95% CI: 0.854–0.888)) and *F*1 score (0.547 (95% CI: 0.539–0.661)) analyses, the extreme gradient boosting (XGBoost) model outperformed the other models (i.e., LGBM, LR, RF, DT, and KNN). Furthermore, SHAP force analysis illustrated how the constructed model visualized the individualized prediction of death. XGBoost machine learning framework gives good in-hospital mortality prediction of elderly patients with sepsis and can maximize prediction model accuracy. The XGBoost model could be an effective tool to assist doctors in identifying high-risk cases of in-hospital mortality among elderly patients with sepsis. This could be used to create a clinical decision support system in the future.

## 1. Introduction

Sepsis is defined as a life-threatening organ dysfunction caused by a dysregulated host response to infection [1]. It is a serious disease with a high mortality rate, and thus, it is considered to be a serious global health problem. In 2017, there were 48.9 million global sepsis cases, and 11 million sepsis-related deaths were reported; these deaths accounted for nearly 20% of all global deaths [2]. Age is an independent risk factor, and the risk of death increases significantly with age [3]. The incidence of sepsis also sharply increases with age [4], and once sepsis occurs in the elderly, there is often a greater risk of death in hospitals [5]. Because the elderly population is among the fastest-growing subgroups of patients admitted to the intensive care unit (ICU), the prediction of sepsis risk is essential for intensive care medicine [6].

There are numerous reasons for why elderly people are more susceptible to infections. Immunosenescence is a condition that is defined as age-related degeneration and dysregulation of immune function; it puts older people at a higher risk of both contracting an infection and developing a more severe and long-term course [7]. Heart failure, chronic obstructive pulmonary disease, malignancies, diabetes mellitus, and chronic liver failure are all prevalent comorbid diseases that raise the risk of infection and subsequent sepsis in elderly patients [8]. In the case of elderly patients with sepsis, their clinical manifestations are atypical because they are prone to a variety of diseases [9]. All of these factors render the diagnosis, treatment, and prognosis of geriatric sepsis challenging, leading to higher mortality. Therefore, early detection or the prediction of high-risk sepsis patients with adverse outcomes can help clinicians to provide appropriate treatment and possibly improve the prognosis of patients, which can critically affect their survival.

Procalcitonin [10], serum lactate [11], albumin [12], and various other biomarkers have been widely used to predict the sepsis-related mortality. However, owing to the clinical heterogeneity of the disease, the accuracy of single biomarker-based prognostication is limited [13]. Establishing prognostic models for patients with sepsis has always been a trending topic in critical care medical research. Such tools include severity scales, which are commonly used to evaluate severity in ICUs; examples include the sequential organ failure assessment (SOFA), systemic inflammatory response syndrome (SIRS) evaluation, and the simplified acute physiology score II (SAPSII) [14–16]. Scoring methods can be relatively simple to implement, as they do not require a lot of information. However, studies have demonstrated that machine learning algorithms outperform scoring methods for ICU patients with extensive and complex clinical data and challenging health assessments [17].

Recently, various machine learning methods have been implemented in the medical field to predict outcomes more accurately. Machine learning models for the early detection of patients at risk of sepsis have been established for ICU [18] and ED [19] settings. Despite the high mortality associated with sepsis or septic shock among elderly patients, machine learning has been often studied in populations older than 18 years or in cohorts not specifically targeting this population but with some older patients enrolled [18–21].

To date, no study has used machine learning to predict the in-hospital mortality of elderly ICU patients with sepsis. Thus, this study is aimed at using the Medical Information Mart for Intensive Care IV (MIMIC-IV) database to develop a valid model for predicting the in-hospital mortality of elderly patients diagnosed with sepsis in accordance with The Third International Consensus Definitions for Sepsis and Septic Shock (i.e., Sepsis-3) [1]. The features were chosen based on their clinical significance and explained in order of priority. This study is in compliance with the transparent reporting of multivariable prediction model for individual prognosis or diagnosis (TRIPOD) reporting checklist [22].

## 2. Methods

### 2.1. Database

Our study was a retrospective cohort study. We used the MIMIC-IV version 1.0 database, which contains data on more than 40,000 ICU patients from Beth Israel Deaconess Medical Center between the years of 2008 and 2019. We carefully studied the course “Protecting Human Research Participants” on the National Institutes of Health website and obtained permission to use the database (certification number: 10264242). The ethics committee at the medical centers did not require informed consent because the private information of patients was encrypted in the database.

### 2.2. Study Population

Our study comprised elderly patients who were diagnosed with sepsis. The criteria for inclusion were as follows: (i) patients who were 65 years or older, (ii) a length of stay in the ICU longer than 24 h, and (iii) patients who were diagnosed with Sepsis-3. According to the Sepsis-3 guidelines, infected patients with a SOFA score of higher than two are classified as having sepsis. We only included the first ICU admission for patients who had two or more ICU admissions during one hospitalization. Lastly, patients whose records had a predictor variable missing rate of more than 40% were eliminated.

### 2.3. Data Extraction and Imputation

We developed structured query language (SQL) scripts with a significant number of SQL statements to query the MIMIC-IV database for elderly sepsis patients. Within 24 h of ICU admission, clinical and chemical characteristics were extracted. The following data from the first day after ICU admission were extracted: age, gender, ethnicity, weight and height on admission, and time of death. Next, we collected the vital signs of the patients, including heart rate, blood pressure, arterial pressure, temperature, respiratory rate, and oxygen saturation. Subsequently, laboratory index data, including the blood routine examination results, liver and kidney function-related data, and arterial blood gas, were withdrawn. Additionally, the life support-related data (mechanical ventilation, renal replacement therapy, etc.) and data on accompanying diseases were extracted. Comprehensive indicators were extracted, such as the SOFA score, SIRS score, Oxford acute severity of illness score (OASIS), logistic organ dysfunction system (LODS), and acute physiology score III (APS III). The baseline aggregation on admission includes laboratory data obtained up to 24 h after ICU admission. For each variable with fewer than 40% missing data, we replaced the missing values by using the K-nearest neighbor (KNN) method.

### 2.4. Statistical Analysis

The statistical analysis was focused on comparing the mortality group to the nonmortality groups. Continuous variable data were evaluated as the mean ± standard deviation under a normal distribution and analyzed by *t*-test. The chi-square test was used to analyze and compare the categorical variables, which were represented as frequencies with percentages. All statistical analyses were performed by using SPSS 25.0 and Python (version 3.9) platforms; the statistical significance was set at *p* < 0.05.

### 2.5. Model Development

To predict in-hospital mortality in elderly patients with sepsis, we applied a machine learning algorithm. We developed six prediction models using extreme gradient boosting (XGBoost), light gradient boosting machine (LGBM), decision tree (DT), KNN, logistic regression (LR), and random forest (RF) algorithms. A grid-search strategy was performed for each model to determine the optimal hyperparameters, with all possible combinations of given candidate hyperparameter values being evaluated. The details of this hyperparameter tuning are provided in Table 1. The hyperparameters that yielded the best values for area under the receiver operating characteristic curve (AUROC) were selected. Finally, all models were compared.

We randomly divided 80% of the MIMIC-IV dataset into a training set at random while reserving the remaining 20% of the dataset as the independent test set. We performed tenfold cross-validation (CV) to validate model performance and minimize the likelihood of overfitting. The training data were split into ten groups, nine of which were used to train the model and one for validation. After cycling through all permutations of the training and validation sets, we then tested each of the ten models on the independent test set. The mean performance metrics were calculated based on the results of these ten models.

A receiver operating characteristic (ROC) curve was used to compare the prediction efficiencies of the models. Model discriminability was tested by using the AUROC. The sensitivity, specificity, positive predictive value, and negative predictive value were also calculated. In addition, we used a Shapley additive explanation (SHAP) algorithm to assess our prediction model, address the matter of black-box predictions, and obtain explanations of the features that drive patient-specific predictions [23]. Finally, we trained and tested the model with the scikit-learn tool.

## 3. Results

### 3.1. Baseline Characteristics

After excluding patients below 65 years of age and those with incomplete clinical data, 18522 elderly patients from the MIMIC-IV database were included in the final analysis, with 15.4% (2845) in-hospital mortality. A flow chart describing the cases is shown in Figure 1. This study included 59 conventional clinical variables. The main characteristics of the elderly patients with sepsis are listed in Table 2.

### 3.2. Model Comparison and Explanation

Table 3 lists the AUROC value, *F*1 score, recall, sensitivity, and specificity findings for each model in tenfold CV for the ideal cut-off position.

Figure 2 depicts the ROC curves for these predictive models. The ROC curve analysis reveals that the XGBoost, LGBM, and LR models could predict in-hospital mortality with a high accuracy and that the results of the XGBoost model were more ideal.

### 3.3. SHAP Values

Figure 3(a) shows the results of evaluating the SHAP values for the XGBoost model. Each row represents a feature. The horizontal coordinate is the SHAP value, the blue color means that the feature's contribution is negative, the red color means that the feature's contribution is positive, and a point represents a sample. Furthermore, a redder color means the feature itself is larger, whereas a bluer color means the feature itself is smaller. This plot shows how high and low feature values in the training dataset are correlated with SHAP values. According to the prediction model, a higher SHAP value for a feature corresponds to a higher likelihood of in-hospital mortality. The APS III, LODS, age, respiration rate, OASIS, maximum red blood cell distribution width (RDW), lowest white blood cell count, lowest lactate, and highest lactate results all indicated a higher likelihood of in-hospital mortality (Figure 3(a)). The significance of these variables was sorted according to their importance value; the results are shown in Figure 3(b). Individual variables were ranked based on their relative influence; the top 20 variables are shown in Figure 3(b).

Finally, as shown in Figure 4, we derived SHAP dependency plots for the first four contributing variables that were applied to explain the impact of the change in value of each variable on the patients' SHAP values. The *y*-axis values indicate the SHAP values for the features, and the *x*-axis presents the range of the original values for the features. Figure 4 illustrates how the attributed importance of the features changed as their values varied. It should be noted that a SHAP value above zero for a specific feature indicates an increased risk of in-hospital mortality development.

## 4. Discussion

In this study, we applied six machine learning models to predict in-hospital mortality in elderly patients with sepsis. The outcome prediction performances of machine learning models on the independent test set were satisfactory. Particularly, the prediction performance of the XGBoost model was superior to those of the other models. Furthermore, the model was elucidated, as we were able to use the SHAP values to explain the variables and describe the effects of their changing trends on the in-hospital mortality.

Recently, machine learning models have been applied for predicting diverse outcomes of sepsis, for example, early identification and prediction [24], clinical phenotype [25], and the occurrence of complications [26]. This big data-driven approach involving the use of an advanced machine learning algorithm has been demonstrated to be superior to traditional analytic models and score models [27]. To the best of our knowledge, this is the first study to predict in-hospital mortality in elderly patients with sepsis based on extensive public data by developing a novel high-performance integrated machine learning model.

We discovered numerous clinical indicators that were linked to a higher likelihood of in-hospital mortality in elderly patients with sepsis. By applying a SHAP value algorithm, we found that the APS III, LODS, age, maximum partial pressure of blood oxygen, and weight of admission were the significant indicators of in-hospital mortality. The APS III [28], LODS [29], and OASIS are commonly used to predict the prognosis of patients with sepsis. Previous studies have shown that these scoring systems can predict the prognosis of septic patients in ICUs better than SOFA or quick SOFA (qSOFA); this is consistent with our findings [30].

In addition to the scoring systems, age was a strong predictor of in-hospital mortality. Below approximately 90 years of age, the significance of age as a predictor of in-hospital mortality clearly showed an increasing trend, particularly for patients above 80 years of age. However, the trend declined for patients over 90 years of age. Previous studies have shown that age is an independent predictive factor for in-hospital mortality for patients aged 80 years and older [4]. Urine output, partial pressure of oxygen (PO_2_), oxygen saturation (SPO_2_), and lactate are the most commonly measured indices; they also play a key role in predicting in-hospital mortality in our study. Humans maintain fluid balance mostly through urinary output, and effective fluid management measures can considerably improve the chances of patient survival [31].

The PO_2_, SPO_2_, and lactate are widely applied as targets of initial resuscitation in patients with severe sepsis and septic shock associated with inadequate tissue perfusion and hypoxia [32]. In our study, the risk of death would be lower for a PO_2_ value below 100 mmHg, suggesting additional benefits by increasing PO_2_ to 100 mmHg. However, increasing the PO_2_ beyond 100 mmHg will negatively impact the likelihood of survival. Several observational studies have demonstrated an association between arterial hyperoxia and increased mortality in different subsets of critically ill patients [33]. A recent systematic review and meta-analysis study demonstrated that a conservative oxygen supplementation strategy was feasible and safe [34].

The significance of the RDW was a fascinating result in our study. The RDW is an erythrocyte index that reflects the heterogeneity in the size of circulating erythrocytes and is used to diagnose or rule out hematological disease. Studies on several clinical conditions, including acute pancreatitis [35], heart failure [36], and pulmonary embolism [37], have recently proved that the RDW is a significant predictor of the outcomes. Researchers previously drew the following conclusions after conducting a comprehensive meta-analysis to assess the prognostic role of the RDW relevance in patients with sepsis; the RDW at baseline is linked to the mortality of patients with sepsis, which could be a simple and valuable prognostic marker for patients with sepsis [38].

Similar methods to predict the mortality risk of patients with sepsis in an ICU setting have previously been applied. In a recent study, Zhang et al. described a random survival forest-based model for 30-day mortality risk predictions for elderly patients with sepsis [39]. They based their model on routinely obtained data, similar to our study. However, they reported that their model did not perform well. In addition, the issue of model interpretability was not discussed. Our model has the benefit of being explainable in terms of the value of individual features for ICU elderly patients with sepsis survival because of the use of SHAP.

The application of such models implies that physicians and caregivers can be notified when an ICU elderly patient's condition becomes complicated with sepsis, thereby affording them time to devise and employ efficient yet individualized therapeutic measures. Although the efficacy of the XGBoost model has been demonstrated, XGBoost is a gradient boosting machine that uses a tree model as a basic weak predictor. We found ensemble-based learning models to be better predictors in previous studies [40, 41]. One of the studies on early prediction of sepsis [42] realized a 6-hour ahead prediction of sepsis using an ensemble framework. They used XGBoost and gradient boosting decision tree as level-2 regressor. Considering ensemble models, it showcased significant improvement (*p* < 0.01) compared with any single model, demonstrating that the ensemble framework is effective for improving predictions. The key to the success of an ensemble model is that individual base learners perform diversely [43]. This approach can enhance the predictive performance of further studies.

Sepsis is common and is associated with high morbidity and mortality. Because of their diminishing physical and functional capabilities, the elderly are more susceptible to contact infection. They have a larger chance of developing sepsis more frequently and with greater severity [8]. It is also known that elderly patients typically have atypical manifestations; thus, they may not have the aberrant vital signs typically seen in septic patients. Given these factors, clinicians may be able to provide an appropriate treatment and improve patient outcomes if individuals at a high risk of developing poor consequences from sepsis are identified early.

### 4.1. Limitations

The study had several limitations owing to its retrospective design. First, the study was performed at a single institution. We require additional data sources to further demonstrate the generalizability of the proposed model. Second, because of the database's limitations, other variables that could have predictive value, such as the serum procalcitonin, C-reactive protein, and blood culture, were excluded from the model because of their extremely high missing rates. This is because of the retrospective character of our study, which limited the completeness of the laboratory data and the availability of the variables needed to calculate the score. Other limitations that are common in retrospective studies, such as potential selection bias, may have existed. Finally, we applied the in-hospital mortality as the primary endpoint, focusing on the all-cause mortality rather than the sepsis-related mortality. This may have resulted in an overestimation of the true sepsis mortality because the corresponding elderly patients may have died from a variety of diseases.

## 5. Conclusions

This study primarily contributes by developing a machine learning-based in-hospital mortality prediction model for elderly ICU patients with sepsis. The evaluation results demonstrated XGBoost as a useful algorithm, with the best predictive performance in predicting in-hospital mortality in elderly patients with sepsis. Model development is currently underway to realize the real-time adjustment of the in-hospital mortality risks of elderly patients with sepsis, as well as use in other clinical outcomes of relevance. These advances will help in optimizing treatment and improving prognosis.

## Figures and Tables

**Figure 1:** Flow chart of the selection process for studied patients.

**Figure 2:** Comparison of the ROC curves for the six models.

**Figure 3:** (a) Feature significance ranking for the feature representation methods of the XGBoost and (b) top 20 features ranking of importance using the SHAP values.

**Figure 4:** SHAP dependency plots of APS III, LODS, age, and maximum PO_2_.

**Table 1:** Hyperparameters and tuning strategies for each model in the study.

Model	Hyperparameters	Grid-search setting
K-nearest neighbors	Number of neighbors	5, 10
	Neighbor weight	Uniform, distance
Decision tree	Maximum depth	10, 50, 100
Random forest	Number of estimators	10, 50, 100
	Maximum depth	10, 50, 100
Logistic regression	Cs	0.1, 1, 10, 100, 1000
LGBM	Learning rate	0.01, 0.1, 1
	Number leaves	5, 10, 15, 20
	Maximum depth	3, 5, 7, 9, 11
XGBoost	Learning rate	0.01, 0.1, 1
	Number leaves	5, 10, 15, 20
	Maximum depth	3, 5, 7, 9, 11

**Table 2:** Baseline characteristics of elderly patients with sepsis.

	Death	Survival	*p*
Number	2845	15677	
Age	77.21 (68.84, 84.76)	74.14 (67.01, 82.24)	<0.001
Male	1537	8818	0.028
Duration of ICU stay	6.67 ± 7.10	4.62 ± 5.94	<0.001
Duration of hospital stay	12.07 ± 14.84	12.03 ± 12.06	<0.001
Scoring systems			
SOFA score	8.97 ± 4.13	5.88 ± 3.17	<0.001
APS III	78.95 ± 27.71	50.74 ± 20.85	<0.001
SIRS score	3.08 ± 0.80	2.84 ± 0.88	<0.001
OASIS	42.03 ± 8.95	34.10 ± 8.46	<0.001
LODS	8.80 ± 3.58	5.28 ± 2.93	<0.001

**Table 3:** Comparison of the performance of the six models.

Model	AUROC	Accuracy	Precision	*F*1 score	Recall
XGBoost	0.871(95% CI: 0.854–0.888)	0.851 (95% CI: 0.842–0.863)	0.503 (95% CI: 0.461–0.611)	0.547 (95% CI: 0.539–0.611)	0.601 (95% CI: 0.585–0.701)
LGBM	0.870 (95% CI: 0.861–0.894)	0.876 (95% CI: 0.868–0.890)	0.654 (95% CI: 0.618–0.735)	0.467 (95% CI: 0.431–0.551)	0.363 (95% CI: 0.317–0.440)
LR	0.857 (95% CI: 0.845–0.881)	0.877 (95% CI: 0.867–0.884)	0.660 (95% CI: 0.627–0.703)	0.48 (95% CI: 0.416–0.525)	0.377 (95% CI: 0.309–0.419)
RF	0.807 (95% CI: 0.795–0.835)	0.866 (95% CI: 0.856–0.875)	0.632 (95% CI: 0.585–0.723)	0.362 (95% CI: 0.318–0.427)	0.253 (95% CI: 0.211–0.303)
DT	0.738 (95% CI: 0.706–0.791)	0.85 (95% CI: 0.836–0.857)	0.5 (95% CI: 0.455–0.555)	0.369 (95% CI: 0.363–0.433)	0.293 (95% CI: 0.272–0.354)
KNN	0.744 (95% CI: 0.682–0.806)	0.857 (95% CI: 0.840–0.875)	0.581 (95% CI: 0.426–0.717)	0.283 (95% CI: 0.254–0.312)	0.187 (95% CI: 0.107–0.267)

## Data Availability

The data utilized to support the findings are available from the corresponding authors upon request. The data applied in the present study were from the MIMIC-IV database (https://mimic.physionet.org/), a freely accessible database.
